The article "Reservoir Physical Properties and Micropore Nanocharacteristics of Cores in the Shihezi Formation, Sudong District, Sulige Gas Field, Ordos Basin" was retracted in 2023. Reasons: signs of a paper mill; compromised peer review; unreliable results or conclusions.

# Reservoir Physical Properties and Micropore Nanocharacteristics of Cores in the Shihezi Formation, Sudong District, Sulige Gas Field, Ordos Basin

**DOI:** 10.1155/2022/6008603

**Published:** 2022-05-13

**Authors:** Xin Zhang, Feng Wang, Shuyi Liang, Qintao Guo, Jingchun Tian, Bingyue Shen

**Affiliations:** ^1^Institute of Sedimentary Geology, Chengdu University of Technology, Chengdu 610059, China; ^2^Dongsheng Jinggong Petroleum Development Group Co., Ltd., Shengli Oilfield, Dongying 257000, China; ^3^Geophysical Research Institute, Shengli Oilfield, Dongying 257000, China

## Abstract

Sulige gas field is a very complex large-scale gas field with low porosity, low permeability, low abundance, and strong heterogeneity. In this study, the nanopore structure of the reservoir in the study area was analyzed. The analysis of reservoir physical properties and core microscopic pore characteristics of Shihezi formation in Sudong District, Sulige gas field, Ordos Basin, was put forward. According to core observation, thin section identification, and grain size analysis, the lithology of gas reservoirs in Shan-1 member and He-8 member in the study area is mainly lithic sandstone, lithic quartz sandstone, and quartz sandstone. According to the analysis of physical data in the study area, the reservoirs in Shan-1 member and He-8 member have typical characteristics of low porosity and low permeability. According to that microscopic observation of sandstone thin section and cast thin section combined with the analysis of scan electron microscope, the results show that both Shan-1 member and He-8 member of Sudong area 2 in Sulige gas field are dominated by class I reservoirs and class II reservoirs. Especially, class I reservoirs are widely distributed, with the cumulative area of this type of reservoirs accounting for 70.12% of the total area in Shan section and 64.12% in He-8 section. Class I reservoirs are scattered in the study area, accounting for 0.27% of the total area in the mountain section and 0.36% in the He-8 section. Class IV reservoirs are distributed dispersedly and have a small distribution area. The cumulative area of reservoirs in mountain section accounts for 5.38% of the total area and that in He-8 section accounts for 5.46%. Therefore, Sudong area 2 in Sulige gas field is a typical low porosity and low permeability reservoir. On the basis of geological background, sedimentary microfacies, diagenesis, and pore structure characteristics of the study area, it is considered that the pore structure of sandstone in the study area is mainly controlled by sedimentary characteristics and diagenesis of sandstone.

## 1. Introduction 

Sulige gas field is located in the northwest of northern Shaanxi slope in Ordos Basin, with an exploration area of 4 × 104km^2^ large-scale continental sandstone lithologic closed gas reservoirs. The research area is the second area of Sudong in Sulige gas field, which is located in the northeast of Sulige gas field. The research horizon is Shan-1 member and He-8 member [1]. The Upper Paleozoic Permian in northern Ordos Basin is characterized by multiple provenances, near provenance, and fast accumulation. The nature of parent rocks in the source area determines the diversity of sandstone types and low compositional maturity in the study area. It also affects the diagenetic evolution and microscopic pore structure characteristics of various sandstone reservoirs and ultimately leads to different development conditions of pores and channels and reservoir properties of various sandstones [1]. Previous studies on the reservoirs in Sudong area 2 of Sulige gas field mainly focused on the macroscopic sedimentary system, petrological characteristics, and diagenesis characteristics, but the pore structure, diagenetic evolution, especially pore evolution of various sandstone reservoirs were not deeply studied [2]. In order to solve this research problem, Xiong M. and others began to study the diagenesis system from different scales (from the basin area to the intralayer area), such as exploring the relationship between small-scale diagenesis characteristics and large-scale basin evolution and thermal fluid activity, thus revealing the temporal and spatial evolution law of diagenesis [3]. Guangfeng L. believed that the dissolution and precipitation of minerals were closely related to the acidity and alkalinity of diagenetic media, and their differences from classical diagenesis were mainly reflected in the following two aspects: on the one hand, the manifestations of alkaline diagenesis mainly included authigenic chlorite film cementation, authigenic illite cementation, rock salt cementation, albitization, carbonate cementation, sulfate cementation, zeolite cementation, and quartz dissolution. On the other hand, early diagenesis stage B was the main pore development stage, while late diagenesis stage A was generally unfavorable to the development of reservoir space [4]. Daniel W used clay, quartz, feldspar, rock cuttings, or modern sediment samples to carry out compaction simulation experiment [5]. Based on this, this study focuses on the in-depth study of pore structure, diagenetic evolution, and pore evolution history of sandstone reservoirs of different rock types in Sudong area 2 of Sulige gas field, which not only has certain theoretical significance. Moreover, it has important practical value for the exploration and development of Upper Paleozoic natural gas in Sudong area 2 of Sulige gas field [6].

The article "Reservoir Physical Properties and Micropore Nanocharacteristics of Cores in the Shihezi Formation, Sudong District, Sulige Gas Field, Ordos Basin" was retracted in 2023. Reasons: signs of a paper mill; compromised peer review; unreliable results or conclusions.

## 2. Methods

### 2.1. Geological Background

Sudong District of Sulige gas field is located in Wushen Banner, Ordos City, Inner Mongolia Autonomous Region, and Yuyang District, Yulin City, Shaanxi Province. The structure is located in the north-central part of Yishan slope in Ordos Basin, showing a west-inclined monoclinal structure with high NE and low SW, and a series of NE-SW nose-uplift structures are developed in it. There are small top bulges and top depressions locally. The provenances of Shan-1 member and He-8 member in Sudong District of Sulige gas field are characterized by a mixture of two provenances [7].

### 2.2. Petrological Characteristics of Reservoirs

According to core observation, thin section identification, and grain size analysis, the lithology of gas reservoirs in Shan-1 member and He-8 member in the study area is mainly lithic sandstone, lithic quartz sandstone, and quartz sandstone, among which the rock types in He-8 member are mainly lithic sandstone and lithic quartz sandstone, with a small amount of quartz sandstone. Shan-1 member is mainly composed of lithic sandstone and lithic quartz sandstone, without quartz sandstone. Rock grain size is generally coarse, mainly medium-coarse sandstone, with the main grain size distribution in the range of 0.2–2.0 mm. The particles are sorted moderately and poorly, and the roundness is mostly subprismatic and round [8].

### 2.3. Reservoir Physical Properties

Porosity and permeability of sandstone reservoir are two basic parameters reflecting reservoir performance and percolation conditions. According to the analysis of physical data in the study area, the reservoirs of Shan-1 member and He-8 member have typical characteristics of low porosity and low permeability. The porosity is low, mainly distributed between 4% and 14% (Figure 1). The average porosity of the He section is 10.31%, the minimum is 4.12%, and the maximum is 17.1%. The average porosity of Shan-1 member is 9.6%, with a minimum of 3% and a maximum of 17.3%. Permeability is mainly distributed in (0.1 − 2) × 10^−3^*μ*m^2^. It can be seen that the distribution of permeability is characterized by double peaks (Figure 2), with the main peak located at the range of (0.3 − 0.4) × 10^−3^*μ*m^2^. The secondary peak is located at 1 × 10^−3^*μ*m^2^. The average permeability of He-8 is 0.57 × 10^−3^*μ*m^2^. The average permeability of Shan-1 member is 0.474 × 10^−3^*μ*m^2^. On the whole, the physical properties of He-8 member are slightly better than those of Shan 1 member [9].

### 2.4. Pore Structure Types

According to the observation of sandstone thin section and cast thin section under the microscope combined with scanning electron microscope analysis, the pore types of Shan-1 member and He-8 member in the study area are mainly secondary pores (secondary dissolved pores, intergranular pores, and cracks), while primary pores (residual intergranular pores) occupy a secondary position [10].

The article "Reservoir Physical Properties and Micropore Nanocharacteristics of Cores in the Shihezi Formation, Sudong District, Sulige Gas Field, Ordos Basin" was retracted in 2023. Reasons: signs of a paper mill; compromised peer review; unreliable results or conclusions.

#### 2.4.1. Residual Intergranular Pore

Affected by compaction and cementation, most of the primary intergranular pores in the study area have disappeared, and only residual intergranular pores have developed locally. Compaction directly reduces the volume of primary intergranular pores, while cementation makes primary intergranular pores filled in different degrees, some diagenetic minerals cause intergranular pores to shrink and pore connectivity to deteriorate. The fillings in the study area are often some terrigenous heterogenous and authigenic clay minerals. As a result of filling, the pores often remain in the form of crevices. The pore size of this kind of pore is generally 5 − 50*μ*m. The proportion in the total pores is small.

#### 2.4.2. Intergranular Dissolved Pore

The intergranular dissolved pores in sandstone in the study area make the edges of dissolved particles very irregular and harbor-like, which have good connectivity and different pore sizes 5 − 50*μ*m.

#### 2.4.3. Intragranular Dissolved Pore

The intragranular dissolved pores in the study area are mainly cuttings dissolved pores and feldspar dissolved pores, and quartz dissolved pores can also be seen. Among them, cuttings dissolution is one of the important contributors to the pores of Shan-1 member and He-8 member in Sudong area 2 of Sulige gas field. Generally, the pore diameter of cuttings dissolution hole is in 50 − 150*μ*m. Local aperture can reach 500*μ*m. The face rate is generally between 0.5% and 1%. Feldspar porosity is also common, but its development degree is not very high, and its contribution to effective porosity of reservoir is generally less than 1%.

#### 2.4.4. Intergranular Pores of Authigenic Minerals

The authigenic mineral intergranular pores in the study area are mainly kaolinite intergranular pores, illite intergranular pores, chlorite intergranular pores, and illite/montmorillonite intergranular pores. This kind of pore radius is small, among which the pore size of kaolinite intergranular pore is 5*μ*m. Kaolinite has a certain connectivity and a large number of pores, which can be effective. Chlorite intergranular pore size is very small, generally less than 1*μm*. It is easy to be saturated by irreducible water and become invalid pores. Intergranular pores are well developed in the sand bodies of Shan-1 member and He-8 member, accounting for about 30% of the total pores, and are one of the important contributors to the pores of the target horizon in the study area.

The article "Reservoir Physical Properties and Micropore Nanocharacteristics of Cores in the Shihezi Formation, Sudong District, Sulige Gas Field, Ordos Basin" was retracted in 2023. Reasons: signs of a paper mill; compromised peer review; unreliable results or conclusions.

#### 2.4.5. Heterogeneous Pore

In the study area, it mainly refers to the dissolved pores formed by the dissolution of mudstone miscellaneous base, which are mostly irregular, and its pore size is often very small, which is not well developed in the study area and has a small contribution value to the effective porosity [11].

#### 2.4.6. Crack

In the process of core observation in the study area, the fracture length of Z59 well, Z72, Z66, and Z65 can be up to 8 m. Most of the fractures are high-angle fractures with a width of 2-3 mm. Most of them are open fractures, and a few of them are half-filled with calcite. Such fractures can increase the permeability of sandstone by 1-2 times and play an important role in transporting oil and gas. This kind of fracture develops well in the study area. Microcracks are mainly distributed in between 5 and 50 *µ*m, and the total porosity is 1-2%. The reservoir space formed by microfractures is very small and has little influence on porosity. However, it is because of the existence of microfractures that the isolated pores are connected to form the infiltration channel of sandstone and improve the permeability of rock [12].

### 2.5. Characteristics of Pore Throat of Reservoir

According to the characteristic parameters extracted from casting thin sections and mercury injection data, the microscopic pore structure characteristics of reservoirs can be quantitatively characterized. The mercury injection method is a commonly used method to study the characteristics of rock pore structure at present, and several important characteristic parameters include parameters reflecting pore throat size: displacement pressure (MPa), median pressure (MPa), median radius (*μ*m), maximum pore throat radius (*μ*m), and average diameter of pore throat (*μ*m); parameters characterizing pore throat sorting: sorting coefficient, variation coefficient, and homogeneity coefficient; and parameters reflecting pore throat connectivity and controlling fluid movement characteristics: maximum mercury inlet saturation (%) and mercury removal efficiency (%). According to the parameter statistical results of capillary pressure measurement in Shan-1 member and He-8 member, the pore structure of sandstone has the following characteristics:

1. From the perspective of pore throat size, member in the study area is characterized by high displacement pressure, low median pressure, and small median radius. The displacement pressure ranges from 0.12–3.84 MPa to 3.84 MPa, with an average of 1.145 MPa, and the median pressure ranges from 1.34 MPa to 35.61 MPa, indicating that the pore throats of rocks are unevenly distributed. The median radius ranges from 0.02 to 0.851 *μ*m, with an average of 0.11 *μ*m. The maximum throat radius is 0.375.65 *μ*m, with an average of 1.914 *μ*m. The median radius is basically less than 0.05 *μ*m. The development of pore throat is the main factor, which reflects that the radius of pore throat in the study area is generally small [13].
2. According to the characteristics of pore throat sorting, the pore throat sorting coefficients of Shan-1 member and He-8 member are between 0.98 and 4.21, with an average of 1.62. The average coefficient is between 0.08 and 0.52, with an average of 0.155. The coefficient of variation is between 0.06 and 0.52, with an average of 0.1351, reflecting the strong diagenesis in the study area.
3. From the perspective of pore throat connectivity, the maximum mercury saturation is distributed in a wide range, ranging from 17.46% to 89.6%, with an average of 65.21%. The mercury removal efficiency is generally ranging from 27.98% to 67.2%, with an average of 53.525%, reflecting the poor pore throat connectivity of Shan-1 member and He-8 member reservoirs [14].

The article "Reservoir Physical Properties and Micropore Nanocharacteristics of Cores in the Shihezi Formation, Sudong District, Sulige Gas Field, Ordos Basin" was retracted in 2023. Reasons: signs of a paper mill; compromised peer review; unreliable results or conclusions.

### 2.6. Pore Structure Characteristics and Evaluation

According to the statistics of pore structure characteristics and mercury injection data, the reservoirs of Shan-1 member and He-8 member in Sudong area 2 of Sulige gas field can be divided into four categories (Figure 3 and Figure 4), in which class I and class II reservoirs are high-quality reservoirs in the study area. Class III reservoirs are medium reservoirs in the study area, and class IV reservoirs are nonreservoirs [15].

#### 2.6.1. Class I Reservoir

The mercury pressure curve is platform type, with good connectivity of pore throat, coarse deviation, low displacement pressure, less than 0.4 MPa, high mercury removal efficiency, and pore throat sorting coefficient less than 1.61. It has good reservoir property, with porosity greater than 12% and permeability generally greater than 1 × 103 *μ*m^2^, which is the best pore structure type in the study area [16].

#### 2.6.2. Class II Reservoir

The mercury pressure curve is a platform type with a constant slope, with good pore throat sorting, displacement pressure of 0.4–0.8 MPa, and median radius of 0.1–0.54 *μ*m. It has good physical properties, with porosity of 9%–12% and permeability of (0.5 − 1) × 10^−3^*μ*m^2^, which is the main pore structure type in the study area.

#### 2.6.3. Class III Reservoir

The mercury injection curve has a large platform slope and good connectivity of pore throat, and the displacement pressure is generally between 0.8 and 2 MPa. The pore combination types are mainly micropore-intergranular pore and dissolved pore-intergranular pore, with medium reservoir properties, porosity of 5%–9%, and permeability of (0.1 − 0.5) × 10^−3^*μ*m^2^. This type of reservoir has medium physical properties and is widely developed in the study area.

The article "Reservoir Physical Properties and Micropore Nanocharacteristics of Cores in the Shihezi Formation, Sudong District, Sulige Gas Field, Ordos Basin" was retracted in 2023. Reasons: signs of a paper mill; compromised peer review; unreliable results or conclusions.

#### 2.6.4. Class IV Reservoir

This kind of pore structure is common in the study area, with steep mercury injection curve, high displacement pressure, generally greater than 2 MPa, low mercury withdrawal efficiency, less than 36.1%, and small median radius. Pore combination types are mainly micropores and micropores-intergranular pores, with poor reservoir physical properties and basically no reservoir capacity. Generally, porosity is less than 5.1% and permeability is less than 0.1 × 10^−3^*μ*m^2^. It is the pore structure type of study area difference [17].

## 3. Results and Analysis

According to the statistical results of mercury injection parameters of all pore structures in the study area, it is concluded that both Shan-1 member and He-8 member of Sudong area 2 in Sulige gas field are mainly class I reservoirs and class II reservoirs, especially class I reservoirs are widely distributed. The accumulative area of this type of reservoir in the Shan-1 member accounts for 70.12% of the total area and 64.12% of the total area in He-8 member. Class II reservoirs are scattered in the study area, and the area of this kind of reservoir accounts for 0.27% of the total area in the Shan-1 member and 0.36% in the He-8 section. Class IV reservoirs are distributed dispersedly and have a small distribution area. The cumulative area of reservoirs in Shan-1 member accounts for 5.38% of the total area and that in He-8 section accounts for 5.46%. Therefore, Sudong area 2 in Sulige gas field is a typical low porosity and low permeability reservoir.

The Permian gas reservoir in Sulige area is sandstone lithologic gas reservoir, and its distribution is mainly controlled by reservoir sand bodies. On the basis of comprehensive analysis of geological background, sedimentary microfacies, diagenesis, and pore structure characteristics in the study area, it is considered that the pore structure of sandstone in the study area is mainly controlled by sedimentary characteristics and diagenesis of sandstone. Sedimentary microfacies have great influence on the spatial distribution and physical properties of reservoir rocks. Different sedimentary microfacies have different rock types, grain sizes, sedimentary structures, lithofacies associations, and original material components. He-8 member in Sudong District of Sulige gas field was mainly formed in braided river-delta sedimentary environment with braided river as the main body. The Shan-1 member was mainly formed in the meandering river-delta sedimentary environment with meandering river as the main sedimentary body, and the lithology deposited in this fluvial sedimentary environment was mainly coarse sandstone, followed by siltstone [18]. Statistics show that grain size is an important factor affecting porosity and permeability of sandstone, especially porosity, and there is a linear positive correlation between grain size and porosity of sandstone. Coarse-grained rocks are often formed in an environment with strong hydrodynamic conditions. In high-energy environment, muddy fillings are difficult to deposit with them, and rocks supported by coarse-grained clastic framework also have high original pore space. The relationship between sandstone physical properties and particle size in the study area is closely related. The statistical results show that porosity is greater than 8.1% and permeability is greater than 0.5 × 10^−3^*μ*m^2^. The median particle size of the reservoir is usually distributed in coarse sandstone above 0.50 mm [19].

The article "Reservoir Physical Properties and Micropore Nanocharacteristics of Cores in the Shihezi Formation, Sudong District, Sulige Gas Field, Ordos Basin" was retracted in 2023. Reasons: signs of a paper mill; compromised peer review; unreliable results or conclusions.

## 4. Conclusion

There are some differences in sandstone characteristics (lithofacies type, particle sorting, and roundness) of different sedimentary microfacies in the study area, which makes the reservoir properties of sandstone different. The study area has been buried for a long time and experienced complex diagenesis. As a result of compaction, the primary intergranular pores between grains are extremely reduced. The slow subsidence rate of Sulige gas field leads to the development of early cementation. Cements such as illite, kaolinite, siliceous, and carbonate account for a large proportion in the study area and have a more serious impact on reservoir physical properties. With the increase of cement content, the porosity and permeability values decrease. Furthermore, the dissolution in the later stage improved the porosity of the reservoir. Volcanism in the same sedimentary period controlled the formation of secondary dissolved pores in reservoirs. The chemical properties of volcanic eruption detritus in fluvial sandy sediments were unstable, and they were easily dissolved to form secondary pores in the middle and late diagenesis stage, which increased the porosity of sandstone.

## Figures and Tables

**Figure 1:** Distribution characteristics of reservoir porosity in the study area.

**Figure 2:** Distribution characteristics of reservoir permeability in the study area.

**Figure 3:** Capillary pressure curve of class I reservoir and class II reservoir.

The article "Reservoir Physical Properties and Micropore Nanocharacteristics of Cores in the Shihezi Formation, Sudong District, Sulige Gas Field, Ordos Basin" was retracted in 2023. Reasons: signs of a paper mill; compromised peer review; unreliable results or conclusions.

**Figure 4:** Capillary pressure curve of class III reservoir and class IV reservoir.

## Data Availability

The data used to support the findings of this study are available from the corresponding author upon request.
